# Identification of the Hub Genes in Alzheimer's Disease

**DOI:** 10.1155/2021/6329041

**Published:** 2021-07-15

**Authors:** Huiwen Gui, Qi Gong, Jun Jiang, Mei Liu, Huanyin Li

**Affiliations:** ^1^Department of Neurology, Minhang Branch, Zhongshan Hospital, Fudan University, 170 Xinsong Road, 201199 Shanghai, China; ^2^State Key Laboratory of Genetic Engineering, School of Life Sciences, Fudan University, Shanghai 200438, China; ^3^Department of General Practice, Minhang Branch, Zhongshan Hospital, Fudan University, 170 Xinsong Road, 201199 Shanghai, China

## Abstract

**Purpose:**

Alzheimer's disease (AD) is considered to be the most common neurodegenerative disease and also one of the major fatal diseases affecting the elderly, thus bringing a huge burden to society. Therefore, identifying AD-related hub genes is extremely important for developing novel strategies against AD.

**Materials and Methods:**

Here, we extracted the gene expression profile GSE63061 from the National Center for Biotechnology Information (NCBI) GEO database. Once the unverified gene chip was removed, we standardized the microarray data after quality control. We utilized the Limma software package to screen the differentially expressed genes (DEGs). We conducted Gene Ontology (GO) and Kyoto Encyclopedia of Genes and Genomes (KEGG) analyses of DEGs. Subsequently, we constructed a protein-protein interaction (PPI) network using the STRING database.

**Result:**

We screened 2169 DEGs, comprising 1313 DEGs with upregulation and 856 DEGs with downregulation. Functional enrichment analysis showed that the response of immune, the degranulation of neutrophils, lysosome, and the differentiation of osteoclast were greatly enriched in DEGs with upregulation; peptide biosynthetic process, translation, ribosome, and oxidative phosphorylation were dramatically enriched in DEGs with downregulation. 379 nodes and 1149 PPI edges were demonstrated in the PPI network constructed by upregulated DEGs; 202 nodes and 1963 PPI edges were shown in the PPI network constructed by downregulated DEGs. Four hub genes, including GAPDH, RHOA, RPS29, and RPS27A, were identified to be the newly produced candidates involved in AD pathology.

**Conclusion:**

GAPDH, RHOA, RPS29, and RPS27A are expected to be key candidates for AD progression. The results of this study can provide comprehensive insight into understanding AD's pathogenesis and potential new therapeutic targets.

## 1. Background

Alzheimer's disease (AD) is typical hippocampal amnesia and cognitive disorder [1]. It is characterized by amyloid plaques (extracellular), neurofibrillary tangles (intracellular), and structural and functional changes in memory-related brain regions [2, 3]. There are about 50 million people with dementia around the world and about 10 million newly emerged diseases annually; 60-70% of these cases are patients with AD. It is shown that the number of people suffering from dementia around the world has increased twofold more from 1990 to 2016. This trend is mainly attributed to the aging and growth of the population [4]. Due to its slow or invisible onset, it is hard to be conscious of its initial. The main manifestations of AD patients include the declined cognitive function, mental and behavioral disorders, and decreased capability of daily living [5]. AD is classified into three stages in view of the deteriorated degree of cognitive capability and physical function [6]. AD devastates numerous people and has become a chief medical and social burden worldwide [7].

As known to all, a variety of complex pathogenic factors, such as genetic and environmental factors, lead to the occurrence of AD [8, 9]. Up to date, it is yet elusive towards the mechanisms involved in AD's pathogenesis, and efficient methods are incomplete to prevent and treat AD [10]. Though several clinical treatments have been applied in combating the cognitive and behavioral deficits associated with AD, they are still needed to be improved due to limitations.

Gene chip technology is a toolset that arranges a large number of nucleic acid molecules in a large-scale array on a small carrier and detects the strength of the hybridization signal by hybridizing with a labeled sample and then determines the number of detected molecules in the sample [11]. It has the advantages of high sensitivity and accuracy, quickness and simplicity, and the ability to detect multiple diseases at the same time [12]. The past decade has witnessed the discovery and validation of more than a dozen of risk genes related to AD. In human prostate cancer, the use of gene chip technology to explore the role of GAB2 in human prostate cancer cells provides a new therapeutic target for prostate cancer [13]. Using lncRNA microarray gene chip technology, it was found that AC002454.1 has a significantly high expression in children with acute leukemia [14], which is related to the immunophenotype and prognosis of children with acute leukemia to a certain extent. Through gene chip technology, it has been identified that miR-937 in peripheral blood mononuclear cells (PBMCs) is involved in the occurrence and development of Kawasaki disease (KD) [15], which provides a new idea for the prevention and treatment of KD coronary artery expansion.

This article is dedicated to screening and identifying the differentially expressed genes (DEGs) in the gene expression profile GSE63061 and DEGs related to AD. We performed function and pathway enrichment analysis of the DEG and subsequently constructed the protein-protein interaction (PPI) network. Finally, we obtained several genes related to AD: GAPDH, RHOA, RPS29, and RPS27A.

## 2. Materials and Methods

### 2.1. Extraction of Microarray Data

The gene expression profile GSE63061 on Illumina HumanHT-12 V4.0 expression beadchip was acquired from the Gene Expression Omnibus (GEO) of NCBI (http://www.ncbi.nlm.nih.gov/gds/) [16]. A total of 112 samples, comprising 72 AD samples and 40 control samples, were studied.

### 2.2. Identifying the DEGs

We utilized the Limma package in R to identify the DEGs, with an adjusted *P* value <0.01. For analyzing the DEGs in-depth, we constructed a heat map utilizing the Pheatmap package (https://cran.r-project.org/package=pheatmap) in R.

### 2.3. Functional Enrichment Analyses for DEG

We performed the enrichment analysis of AD-associated genes by Gene Ontology (GO) and the Kyoto Encyclopedia of Genes and Genomes (KEGG) analyses utilizing the Database for Annotation, Visualization and Integrated Discovery (DAVID; https://david.ncifcrf.gov/tools.jsp) [17]. GO terms containing biological processes, molecular functions, and cellular components could commendably illustrate the biological function for identified DEGs. As a public encyclopedic database, KEGG comprehensively analyzed the function and biochemical pathways of selected DEGs. If *P* < 0.05, the result is considered statistically significant.

### 2.4. PPI Network Analysis of DEGs

We employed the STRING database (http://string-db.org) [18], which was applied for the Retrieval of Interacting Genes to construct the PPI network. To dig out AD-associated hub protein and key genes, we obtained the interaction between DEGs with a total score ≥ 0.4 and then constructed a PPI network utilizing the STRING database. Finally, we conducted the Cytoscape software to visualize the network and uncover hub genes with higher degrees (connected nodes) in the PPI network. These genes might have a vital role in the network.

## 3. Result

### 3.1. Identification of DEGs in AD

All the blood of AD patients and healthy people from the datasets (GSE63061) was used for our research. We firstly analyzed the DEGs between AD samples and age-matched normal samples. We obtained 2169 genes. The genes with the most significant *P* values are RPL36AL, LOC100132795, NDUFA2, and so on. Then, we utilized a heat map of identified DEG in the GSE63061 database to conduct cluster analysis (Figure 1). Genes with upregulation and genes with downregulation were shown as red and green, respectively. 1313 DEGs were indicated as genes with upregulation, and 856 DEGs were indicated as genes with downregulation.

### 3.2. GO and KEGG Enrichment Analyses

To obtain the function and pathway of these DEGs, we used the online tool DAVID to analyze 1313 upregulation DEGs and 856 downregulation DEGs. Functional enrichment analysis showed that these DEGs with upregulation exhibited a significant association with the immune response of activated neutrophil involvement, the degranulation of neutrophils, and the immunity mediated by neutrophils (Figure 2(a)). Lysosome, osteoclast differentiation, and phagosome were significant pathway enrichment of these upregulated genes (Figure 2(b)). The DEGs with downregulation were mainly related to peptide biosynthetic process, translation, ribosome, and SRP-dependent cotranslational protein targeting to the membrane (Figure 3(a)). Ribosome, oxidative phosphorylation, and nonalcoholic fatty liver disease (NAFLD) were significant pathway enrichment of these DEGs with downregulation (Figure 3(b)).

### 3.3. PPI Network Analysis

We carried out a PPI network analysis to explore the interaction and hub genes of DEGs. Except for disconnected nodes in the network, 379 nodes (proteins) and 1149 PPI edges (interactions) were demonstrated in the PPI network constructed by upregulated DEGs (Figure 4). Likewise, 202 nodes (proteins) and 1963 PPI edges (interactions) were observed in the PPI network constructed by downregulated DEGs (Figure 5). Considering the information of the STRING database, we have chosen the top node with a higher node degree. The number of edges was positively correlated with the importance of their function in the PPI network. The edges and nodes of the connecting lines of these genes were very dense. Among the genes with upregulation, GAPDH and RHOA were thought of as hub proteins and key genes. Among the genes with downregulation, RPS29 and RPS27A are the most important. This suggests they might play an important function in AD development.

## 4. Discussion

As an intricate and refractory neurodegenerative disease, AD seriously affects people's life and living quality, particularly for the elderly [19, 20]. Its pathogenesis is not yet clear, and no effective cure has been developed [21]. Thus, AD is still a major problem in human diseases. Many hypotheses explain the pathogenesis of AD, including amyloid cascades, hyperphosphorylation, neurotransmitters, and oxidative stress [22, 23]. However, the root cause and optimal treatment plan are still difficult to achieve. Xia et al. found out DEGs from the single-cell microarray data of four brain regions affected by AD and constructed a PPI network [24]. Analysis shows that the increase of oxidative stress and the changes in neuronal lipid metabolism may be some events that occur in the early stage of AD pathology. Lee et al. pointed out that p38MAPK could mediate a variety of AD-associated events, i.e., the phosphorylation of tau, neurotoxicity, neuroinflammation, and the dysfunction of synapsis. Therefore, inhibiting p38MAPK is a prospective treatment for AD [25]. Kajiwara et al. believe that the expression of caspase-4 in microglia is related to cognitive impairment in AD [26]. Further research on caspase-4 will be beneficial for comprehending AD's etiology and uncovering new targets for treating AD. Therefore, identifying the key genes involved may help to further understand the development of Alzheimer's disease.

We used public databases to identify and screen DEGs and related pathways in AD through various bioinformatics methods. We identified GAPDH, RHOA, RPS29, and RPS27A as the hub proteins and key genes of AD. Previous studies have shown that GAPDH is a regulator of cell death, and GAPDH is involved in tumor progression and has become a new therapeutic target. Research by Hwang et al. showed that GAPDH-mediated mitosis eliminated defective mitochondria and led to apoptosis, which can provide a potential treatment method for the treatment of Huntington's disease and other neurodegenerative diseases [27]. Mirabello et al. pointed out that RPS29 was a constituent of the small 40S ribosomal subunit which functions essentially in rRNA processing and ribosomal biogenesis and also reported that RPS29 could cause autosomal dominant Diamond-Blackfan anemia [28]. Researchers have shown that RPS27A may be a potential target of mesenchymal stem cells in treating type 2 diabetes mellitus (T2DM).

Functional enrichment analysis revealed that DEGs with upregulation primarily took part in and were enriched in the immune response, neutrophil degranulation, lysosome, osteoclast differentiation, and so on. Mishra and Brinton's research has pointed out that the inflammatory immune response is the unifying factor that connects each risk factor of AD [29]. The DEGs with downregulation exhibit a significant enrichment in peptide biosynthetic process, translation, ribosome, and oxidative phosphorylation. Beck et al. pointed out that reducing mitochondrial oxidative phosphorylation could lead to defects in AD, and mitochondrial dysfunction was one of the early manifestations of AD [30].

This study has some limitations. First, the key DEGs need to be verified by RT-qPCR. In future studies, we will collect clinical samples to verify the expression levels of key DEGs through RT-qPCR. Secondly, we plan to further explore the mechanism of key genes in AD in the animal model.

## 5. Conclusion

In summary, we identified 2169 DEGs between AD patients and healthy controls. Functional enrichment analysis demonstrated that DEGs with upregulation displayed a significant association with immune response, neutrophil degranulation, lysosome, and osteoclast differentiation; the DEGs with downregulation exhibited a significant association with peptide biosynthetic process, translation, ribosome, and oxidative phosphorylation. Subsequently, we identified GAPDH, RHOA, RPS29, and RPS27A as key genes in AD by analysis of the PPI network. The purpose of this research is to improve our understanding of the molecular mechanism of AD through comprehensive bioinformatics analysis and may give a hint of developing the treatment of AD patients.

## Figures and Tables

**Figure 1:** Heat map analysis of identified DEGs between AD specimens and healthy controls. The genes with upregulation and downregulation were indicated as red and green, respectively.

**Figure 2:** Biological process (BP) and KEGG analysis for the DEGs with upregulation. (a) BP analysis and (b) KEGG pathway analysis.

**Figure 3:** Biological process (BP) and KEGG analysis for the DEGs with downregulation. (a) BP analysis and (b) KEGG pathway analysis.

**Figure 4:** The PPI networks were established by significant DEGs with upregulation, which is composed of 379 nodes and 1149 PPI edges. Nodes mean proteins, and edges mean the interaction of proteins.

**Figure 5:** The PPI networks were established by significant DEGs with downregulation, which is composed of 202 nodes and 1963 PPI edges. Nodes mean proteins, and edges mean the interaction of proteins.

## Data Availability

The datasets used and/or analyzed during the current study are available from the corresponding author on reasonable request.
